The article "Quantifying the Dynamic Stability of Gait Patterns in People with Hallux Valgus" was published in 2021. Journal: Appl Bionics Biomech.

# Quantifying the Dynamic Stability of Gait Patterns in People with Hallux Valgus

**DOI:** 10.1155/2021/5543704

**Published:** 2021-05-10

**Authors:** Chaneun Park, Nyeonju Kang, KyoungKyu Jeon, Kiwon Park

**Affiliations:** ^1^The Department of Mechatronics Engineering, Incheon National University, Republic of Korea; ^2^Division of Sport Science & Sport Science Research Institute, Incheon National University, Republic of Korea

## Abstract

Hallux valgus (HV), which is mainly caused by the wearing of narrow-width and high-heeled shoes, disrupts gait behavior because it deforms lower limb joints. There is limited information regarding the relationship between the foot disease HV and lower limb joints. Previous studies evaluating abnormal gait patterns caused by deformity used spatiotemporal parameters; however, they failed to characterize the overall gait dynamics. To address this issue, this study is aimed at characterizing the gait stability of patients with HV and examining the joints that are critically affected by HV. To assess complex gait dynamics, we quantified the potential changes in gait stability by using the maximum Lyapunov exponent (MLE). Angular displacements of the ankle, knee, and hip in the sagittal plane during walking were investigated to calculate the MLE for gait stability based on foot conditions (i.e., barefoot, flat shoes, and high heels). During walking, a large MLE (*P* < 0.05) was noted for the knee joints of subjects with HV, relative to the other lower limb joints. HV appears to have the most critical effect on the knee joints during walking. Ankle movement exhibited higher dynamic stability than the other joint movements of the lower limb (*P* < 0.05). The type of shoe used in the experiment showed no significant dependence with gait stability and joint movement (*P* > 0.05). Quantitative assessments of dynamic stability using the MLE may help clinicians assess the overall gait dynamics of HV patients and other people suffering from gait disturbances.

## 1. Introduction

Hallux valgus (HV) is a foot disease that is mainly caused by constrictive footwear; it has a high incidence rate in women who frequently wear high-heeled shoes. Due to HV, the angles between the metatarsal bones exceed 15°, and the big toe is abducted away from the longitudinal axis of the foot [1, 2]. HV is related to several aspects such as genetic factors, foot structure, sex, age, and shoes [3, 4]. Furthermore, if the big toe joint is congenitally bent or an individual has flat feet, the likelihood of HV increases. Recent studies have suggested that shoes play a potential role in the development of HV [5–7]. Among the various shoe types, narrow shoes with high heels result in excessive pressure being applied on the big toe, which increases the probability of HV; such shoes also increase the impact load during walking. Moreover, increased knee flexion at the heel strike and during the stance phase is observed when wearing high-heeled shoes. Clinically, HV is more likely to occur in women and older people [2, 8, 9].

The article "Quantifying the Dynamic Stability of Gait Patterns in People with Hallux Valgus" was published in 2021. Journal: Appl Bionics Biomech.

Previous studies have associated HV with foot pain, negative effects on body balance and gait patterns, and an increased risk of falls [10–13]. Furthermore, the deformation in the shape of the foot, caused by HV, affects the gait pattern. HV patients alter their gait pattern by moving the central axis of the body outward due to the pain in their big toe [14]. Typically, the lower limb joints are organically connected and move in a complex manner during walking [15]. However, this is disrupted by HV, a foot disease that is likely to affect the lower extremities. Despite this, the relationship between HV and the lower limb joints has not been investigated thoroughly.

A majority of the previous studies on gait stability have characterized human gait using a single gait parameter. For the gait stability of HV patients, gait parameters such as stride, cadence, pressure, and step length have been compared [16–18]. However, it is difficult to elucidate the characteristics of human gait, which can be spatiotemporally complex, using data pertaining to a single variable [19]. Gait stability can be estimated by measuring the changes in variability with respect to time and various dimensions [20]. Kinematic variability alone cannot completely explain dynamic stability [21, 22]. Therefore, to quantitatively assess gait parameters, nonlinear dynamics analysis tools are applied to human gait datasets.

The maximum Lyapunov exponent (MLE), one such nonlinear dynamics analysis method, estimates the local stability of a system [21, 23, 24]. The MLE can be used to represent gait stability by quantifying the ability of the human dynamic system to attenuate small perturbations in the gait trajectory that occur over time [25–29]. For example, people without neurological diseases or musculoskeletal disorders use their body to dampen variability and improve gait stability, in order to maintain a stable gait pattern even in situations involving disturbances. A larger MLE results in faster divergence and indicates lower dynamic stability [21]. The MLE has also been used to investigate gait stability of specific groups, such as the elderly and patients with knee arthritis [1, 25].

In this study, considering shoes as a cause of HV, the relationship between the type of shoe and gait stability was investigated. To overcome the shortcomings of previous research, this study is aimed at (1) estimating the gait stability of people with HV based on foot conditions by using the MLE and (2) investigating the effects of HV on the dynamic stability of the movement of the lower limbs. Specifically, this study focused on determining and examining the joints that are most critically affected by HV. We hypothesized that the movement of the ankle joint, which is closest to the foot, would be more unstable during walking, as compared to the movement of other lower joints, such as the knee and hip joints.

The article "Quantifying the Dynamic Stability of Gait Patterns in People with Hallux Valgus" was published in 2021. Journal: Appl Bionics Biomech.

## 2. Materials and Methods

### 2.1. Data Collection

Fourteen middle-aged women with HV participated in this study. These participants with HV exhibited a moderate degree of deformity (the angle between the metatarsal bones ranged from 20° to 40°). The average age of the participants was 58 ± 11.33 years; the average height was 160 ± 6.73 cm, and the average body weight was 58 ± 5.02 kg. The experiments conducted in this study were approved by the institutional review board of Incheon National University. All the participants provided written consent and voluntarily agreed to participate in the study.

Eight cameras (Motion Analysis Corp., USA) were placed at a distance of approximately 5 m from the subject. Subsequently, calibration was performed to determine the spatial coordinates that fully covered the subject's motion during the experiments. The sampling rate was set at 120 frames per second. To collect three-dimensional data of the human body, 19 reflective markers with a diameter of 10 mm were attached around the pelvis and the lower limbs of the participants, according to the Helen Hayes Marker Set. Kinematic data pertaining to the treadmill walking of each participant were obtained.

The subjects were instructed to wear the shoes provided and walk according to the following conditions, respectively: (1) barefoot, (2) while wearing flat shoes with 1 cm high heels, and (3) while wearing 5 cm high heels. For the experiment, the subjects walked on a treadmill (Apsun Inc., Korea) at their preferred speed. The participants were instructed to walk at their preferred speeds for each condition in order to avoid unusual gait patterns.

Prior to data collection, the experimental procedures and methods were explained to the participants for approximately 10 min. Moreover, the participants were allowed to walk and familiarize themselves with the shoes used for the experiment. Initially, while the participants stood on the treadmill, a researcher adjusted the speed of the treadmill until the preferred speed was reached; the preferred speeds were determined by decreasing or increasing the current speed by fixed steps of 3.5 m/s. The average preferred speed for all shoe conditions was found to be 3.91 ± 0.41 m/s. After the participants' practice, the experiment on the treadmill was commenced. For each foot condition, after 30 s of warm-up, the participants walked at their preferred speed for 30 s. In each trial, the three foot conditions were tested. Between these conditions, the participants were allowed a break of a maximum of 5 min, if they needed one. A total of three random order trials were conducted, each involving the three shoe conditions (i.e., barefoot, flat shoes, and high heels) [30].

The article "Quantifying the Dynamic Stability of Gait Patterns in People with Hallux Valgus" was published in 2021. Journal: Appl Bionics Biomech.

### 2.2. Maximum Lyapunov Exponent Implementation

Dynamic stability can be estimated using the Lyapunov exponent [11, 28]. The average logarithmic divergence rate for extremely close trajectories was quantified using the MLE in a reconstructed state space. During walking, the human body can be considered as a nonlinear system, where the initial state is altered to a completely different state over time [4]. The Lyapunov exponent is a variable that quantifies the distance between two points in proximity as they move away over time [24]. For the Lyapunov exponent, the small perturbations arising from the difference between stride lengths are traced [22]. A Lyapunov exponent exists for each moving dimension in the analyzed gait trajectory. When the divergence rate is high, the Lyapunov exponent has the highest value; this value is called the Maximum Lyapunov Exponent, i.e., *λ*_max_ [20, 24]. Data were analyzed without filtering and resampling to accurately represent the variability within the system. Kinematic data pertaining to the lower extremity of each subject were analyzed to obtain the time series data over 30 gait cycles [22].

The time series data collected through the experiment form a one-dimensional column vector. The acquired kinematic data (i.e., those of the joint angles in the lower extremity: hip, knee, and ankle) are necessary for reconstructing the time series into an *m*-dimensional state space in order to determine the ideal dynamic disturbance based on the joint angle. The time delay method was used to reconstruct the air tractor from scalar data to the *𝓂*-dimensional state space. State-space reconstruction via time-delay methods is sensitive to the delay time [13]. Various methods for determining the time delay, *T*_*d*_, exist; however, the optimal method has not been identified. To ensure that all the experimental data were analyzed under identical conditions, a constant time delay of 10 was used for all the reconstructed state spaces (Figure 1(a)). This time delay is sufficiently sensitive for determining the success of state-space reconstruction. In most previous studies, the time delay was set to 10% of the gait cycle.

The article "Quantifying the Dynamic Stability of Gait Patterns in People with Hallux Valgus" was published in 2021. Journal: Appl Bionics Biomech.

A priori knowledge or definite criteria for determining the embedding dimension do not exist. Therefore, the best approach is to set various embedding dimensions and attempt to determine the value of *𝓂*. Satisfactory results can only be obtained if *𝓂* is at least as large as the topology dimension *𝓃*. This is because the confusion system is probabilistically effective when constructed to accommodate the dynamics of a small phase space. Therefore, choosing the smallest embedded dimension that affords the most satisfactory results is important [22].

The data of each row (*H*_*i*_) of the reconstructed attractor **H** are represented by a matrix, where each row is a phase space vector. An attractor is a set of numeric values that the system tends to evolve for various starting conditions of the system. In a finite-dimensional system, an attractor is an area of *n*-dimensional space if it can be represented as an *n*-dimensional vector.

(1) $$\begin{array}{c} H=\left[\begin{array}{c} H_{i}\\ H_{i+1}\\ H_{i+2}\\ \vdots \\ H_{i+N} \end{array}\right]=\left[\begin{array}{c} \begin{array}{c} h_{i}\;h_{i+T_{d}}\cdots h_{i+\left(m-1\right)T_{d}}\\ h_{i+1}\;h_{\left(i+1\right)+T_{d}}\cdots h_{\left(i+1\right)+\left(m-1\right)T_{d}}\\ h_{i+2}\;h_{\left(i+2\right)+T_{d}}\cdots h_{\left(i+2\right)+\left(m-1\right)T_{d}} \end{array}\\ \vdots \\ h_{i+N}\;h_{\left(i+N\right)+T_{d}}\cdots h_{\left(i+N\right)+\left(m-1\right)T_{d}} \end{array}\right], \end{array}$$

where *h*_*i*_ constitutes the time series data of the joint angles, *T*_*d*_ is the time delay or reconstruction delay, *𝓂* is the embedding dimension for creating an *𝓂*-dimensional state space, and *N* is the number of the time series.

The MLE was calculated based on the Rosenstein algorithm, which is simple and quick in terms of implementation, because it uses simple exponential divergence measurements. Moreover, all available data can be leveraged to correlate small datasets, without requiring large datasets [24].

After the attractor is reconstructed according to the Rosenstein algorithm, the nearest neighboring point of each point in the phase trajectory should be identified in the nearby trajectory, except for the same trajectory. The Euclidean distance *d*_*j*_(*t*) between the closest neighbors was calculated for each data point *i* in the reconstructed state space *d*_*j*_(*t*) for time *t*. The nearest neighbors were found near the nearest data point in a cycle separated from the reconstructed attractor (Figure 1(b)).

(2) $$\begin{array}{c} p\left(i\right)=\frac{1}{i∆t}\ln d_{j}\left(i\right). \end{array}$$

If all the trajectories during walking are identical, the distance between the closest neighbors will be zero. However, after reconstructing the collected time series data into multiple dimensions, the distance between the closest neighbors appears to exceed zero. The changes in the distances between nearest neighbors over time can be estimated from the obtained kinematic data.

The article "Quantifying the Dynamic Stability of Gait Patterns in People with Hallux Valgus" was published in 2021. Journal: Appl Bionics Biomech.

In Eq. (2), the slope of the log of the average divergence becomes the MLE (Figure 2). Positive values of the MLE indicate that the gait trajectory tends to diverge around the average; such values represent a less stable pattern. The larger the value of the MLE, the lower is the stability of the gait pattern. When the value of the MLE is less than or equal to zero, the gait pattern can be considered as a stabilized gait stride in which, on average, extremely close trajectories do not diverge.

### 2.3. Statistical Analysis

A quantitative comparison of gait stabilities was performed via ANOVA using SPSS (Statistical Package for the Social Sciences, Chicago, IL, U.S.A.), with a significance level of *P* < 0.05. Significant differences, as indicated by the analyses, were assessed post hoc using Bonferroni's test. A two-way repeated-measures ANOVA was used to assess the within-participant effects of the joints and shoe types on the value of *λ*_max_.

## 3. Results

Gait stability was quantified by using all the kinematic data and was determined using the MLE values for each lower limb joint. The *λ*_max_ values showed a statistically significant difference (*P* < .05) for the respective joint motions (Figure 3(a)). The mean value of *λ*_max_ was 0.049 ± 0.01 for the ankle, 0.057 ± 0.01 for the knee, and 0.054 ± 0.01 for the hip. Post hoc analyses demonstrated that the value of *λ*_max_ for the ankle was significantly lower (*P* < .05) than those for the hip and knee. Moreover, *λ*_max_ for the hip was significantly lower (*P* < .05) than that for the knee. These values are listed in Table 1.

The *λ*_max_ values showed no significant dependence (*P* > .05) on the foot conditions considered in this study (Figure 3(b)). The mean value of *λ*_max_ was 0.053 ± 0.01 for the barefoot case, 0.053 ± 0.01 for the flat shoe case, and 0.053 ± 0.01 for the high-heel case. The comparison of the mean *λ*_max_ in the foot condition for the different joints also showed no significant differences (Figure 4).

## 4. Discussion

Using the MLE, we have sought to assess the dynamic stability of the joints of people with HV during walking. Little is known about which of the lower extremity joints in HV patients are most critically affected. This study is aimed at quantifying gait stability using the kinematic data of the lower limb joints and at determining and investigating the joint on which HV has the greatest effect. Kinematic data of the joints in the lower extremity, obtained during the walking experiment, were numerically analyzed based on the foot condition. Further, the quantified values were compared to identify significant differences. Specifically, in this study, the differences in dynamic stability of the three joints (ankle, knee, and hip) are provided as quantified values using MLE.

The article "Quantifying the Dynamic Stability of Gait Patterns in People with Hallux Valgus" was published in 2021. Journal: Appl Bionics Biomech.

The higher MLE values at the knee joint showed that, for people with HV, the lowest local dynamic stability is observed at the knee joint, as compared to that at the lower limb joints. This implies that HV has a critical effect on the knee movements. Studies have shown that people with HV also suffer from a high incidence rate of secondary diseases such as knee osteoarthritis; the findings suggest that the knee joint becomes unstable [15, 31]. A previous study reported that wearing high-heeled footwear increases knee movement, resulting in a wide range of movements during walking [32, 33]. Specifically, the knee movements of HV patients who had been wearing high heels for a long time exhibited large differences in motion trajectory between strides. Although HV is a foot disease, it may necessitate orthopedic treatments related to the knee joints.

The MLE of the ankle was the lowest, compared to that of the hips and knees. A lower MLE indicates higher walking stability; in other words, a repetitive pattern of the ankle joints is observed during walking. When wearing high heels, the length of the ankle's periosteum is reduced, whereas the size and stiffness of the Achilles tendon are increased [34]. This reduces the range of movement of the ankle during high-heeled walking [17, 35]. This finding supports the observations in this study; that is, lower MLE values are noted due to lower ankle flexibility because of the severe deformation caused by HV. Moreover, this is different from our initial hypothesis that the ankle would exhibit unstable patterns during walking.

There was no significant difference in the MLE for the three foot conditions considered in the experiment; the three shoe types had no effect on joint motion. In this study, the participants had worn high heels for decades; therefore, they were able to create consistent gait trajectories when wearing the shoes. As the joint was already deformed, a difference in the height of the heel did not appear to have a significant effect on the movement of the joint. Thus, in terms of the MLE, which examines small perturbations in the gait trajectory, the type of shoe had little impact on joint motion.

The article "Quantifying the Dynamic Stability of Gait Patterns in People with Hallux Valgus" was published in 2021. Journal: Appl Bionics Biomech.

This study had a few limitations. Here, gait stability was quantified and estimated with data obtained through experiments involving treadmill walking. Thus, the MLE values may be slightly lower than those for walking on the ground. Furthermore, fixed-speed treadmills cannot help recreate an individual's gait pattern on the ground. Previous studies have suggested that treadmills can artificially reduce natural variability and improve the dynamic stability of gait patterns [22, 36]. Nevertheless, the comparisons presented herein are valid, because dynamic stability was quantified using data from the same treadmill at the rate preferred by each participant. Clearly, if these subjects were to walk on the ground and the study repeated, slightly different MLE values may be generated. Nevertheless, the differences in joint stability are expected to remain the same. Another limitation is that the gait experiment was not conducted randomly. Prior to the experiment, participants were allowed to familiarize themselves with the shoes used in the experiment. As all the participants suffered from HV and were assigned the same type of shoes during the experiment, the experimental conditions can be considered identical, albeit they might have affected the results.

## 5. Conclusions

This study characterized the gait behavior of people with HV and determined the lower extremity joints that were most affected by HV. To quantitatively investigate how HV affects gait stability, the MLE was applied to kinematic data of the lower extremities. MLE analyses showed that HV had the most significant effect on the knee joint when walking, relative to the other lower limb joints. Specifically, the movement of the knee exhibited a large difference in motion trajectory between strides and decreased dynamic stability during walking. Ankle movement showed relatively higher dynamic stability than the other joints of the lower limb. This may be attributed to the long-term decrease in the range of motion of the ankle joint caused by wearing high heels, a factor increasing the probability of HV. Clinicians can apply the observations of this study to examine the overall gait dynamics of people with other gait disorders that are yet to be investigated thoroughly.

## Figures and Tables

**Figure 1:** Schematic of divergence of the nearest neighboring trajectories in the reconstructed attractor. (a) Attractor reconstructed by delaying time series data by a time delay (*T*_*d*_) and three embedded dimensions. (b) Euclidean distance (*d*_*j*_(*t*)) in the reconstructed attractor.

**Figure 2:** Average logarithmic divergence over time.

**Figure 3:** Average maximum Lyapunov exponent (*λ*_max_) with SD for (a) joint angles of lower limbs and (b) three different foot conditions. Capital letters denote significant difference from indicated other lower limb joint (A: ankle; K: knee; H: hip).

The article "Quantifying the Dynamic Stability of Gait Patterns in People with Hallux Valgus" was published in 2021. Journal: Appl Bionics Biomech.

**Figure 4:** Comparison of the average *λ*_max_ under the foot conditions, for the different joints.

**Table 1:** Mean maximum Lyapunov exponent (SE) and *post hoc* analyses of lower limb joints. A superscript letter denotes significant difference from the indicated other lower limb joint.

	Lower limb joint mean (SE)		
MLE	Ankle (A)	Knee (B)	Hip (C)
	0.054^BC^ (0.00083)	0.057^AC^ (0.00025)	0.049^AB^ (0.00023)

*P* value		≤0.001	
*F*		0.3	
*η* ^2^		0.04	

## Data Availability

The experiment data used to support the findings of this study are available from the corresponding authors upon request.
